# He's Yangchao Recipe Ameliorates Ovarian Oxidative Stress of Aging Mice under Consecutive Superovulation Involving JNK- And P53-Related Mechanism

**DOI:** 10.1155/2022/7705194

**Published:** 2022-07-08

**Authors:** Ying Zhao, Yun Chen, Chenyun Miao, Ruye Wang, Liuqing Yang, Jingjing Liu, Zhongfang Chen, Qin Zhang, Jing Ma

**Affiliations:** ^1^Zhejiang Chinese Medical University, Hangzhou 310053, China; ^2^Hangzhou Hospital of TCM Affiliated to Zhejiang Chinese Medical University, Hangzhou 310007, China; ^3^State Key Laboratory of Subtropical Silviculture, Zhejiang A & F University, Hangzhou 311300, China

## Abstract

**Objective:**

To evaluate the effects of He's Yangchao Recipe (HSYC) on ameliorating ovarian oxidative stress of aging mice under consecutive superovulation.

**Methods:**

An 8-month-old C57BL/6 female mouse was chosen to establish an aging model under ovarian hyperstimulation. Mice were randomly separated into four groups: *R*1 as the control group, *R*4 as the model group, NR4 with N-acetyl-L-cysteine (NAC) administration, and TR4 with HSYC administration. Oocyte collection, in vitro fertilization, and embryo culture were performed. The serum hormone levels were measured by enzyme-linked immunosorbent assays (ELISA); the reactive oxygen species (ROS) level of oocytes, the number of growing follicles, corpus luteum, ovulated oocytes, and developing embryos at each stage, along with the proportions of fragmented oocytes and abnormal mitochondria in granulosa cells (GCs) and the apoptosis rate of GCs were calculated; the mRNA and protein levels of JNK, P53, BAX were detected by real-time PCR and the Simple Western System.

**Results:**

HSYC enhanced estradiol, progesterone, and inhibin-B levels and increased growing follicle and corpus luteum and ovulated egg counts compared to the *R*4 group (*P* < 0.05), whereas it decreased the proportions of fragmented oocytes (*P* < 0.01); Meanwhile, embryos from mice subjected to four superovulation cycles with HSYC treated had a higher hatching potential. The ROS level of oocytes is downregulated by HSYC (*P* < 0.01) and the percentage of abnormal mitochondrial in ovaries of the TR4 group was also significantly declined compared to the R4 group (*P* < 0.05); the most TUNEL-positive cells proportion was detected in the *R*4 group; nevertheless, HSYC effectively attenuated this detrimental effect (*P* < 0.05). The mRNA and protein expressions of JNK and P53 in ovary tissues were reduced in the TR4 group while these genes were upregulated by repeated superovulation (*P* < 0.05).

**Conclusions:**

HSYC exerted promising effects on promoting the diminished ovarian reserve and decreased oocyte quality induced by both aging and consecutive ovarian superovulation, potentially via the ROS/JNK/p53 pathway.

## 1. Introduction

Aging, a hotspot arising intense discussion, is considered the main trigger that causes gradual depletion of ovarian reserve and a reduced ability to produce oocytes competent for fertilization in females. Altogether with a progressive reduction of the follicles, woman aging also involves a compromised competence of the embryos [1]. A large retrospective study showed that females over the age of 42 had a live-born baby rate of only 1%, but those under 35 had a rate of 26% [2]. The aging phenomena can be attributed to increased reactive oxygen species (ROS) levels and cumulative oxidative stress in somatic cells [3, 4]. Moreover, mitochondria are the most remarkable targets of ROS, and the dysfunction of mitochondria would induce nondisjunction of the chromosomes, gestation failure, and decreased embryonic viability [5, 6].

Procedures for superovulation and assisted reproductive technologies (ART) are highly successfully and widely used as clinical approaches to treating couples with infertility issues. Though repeated superovulation is considered safe, previous studies have demonstrated that it has some detrimental effects on female reproduction. Several studies showed that ovarian hyperstimulation can lead to pregnancy loss and delayed puberty in female offspring, decreased serum hormone levels, impaired mitochondrial function in ovarian cells, and reduced the oocyte and embryo quality [7–10].

Nowadays, the number of elderly women seeking ART help is gradually increasing. One research studying the intrinsic fertility of the human oocyte showed that natural cycles have higher intrinsic fertility per oocyte than hyperstimulated cycles [2]. It's also been reported that in *in vitro* fertilization (IVF), maternal age is among the strongest predictors of success [11].

It has been demonstrated that traditional Chinese medicine (TCM) is a promising alternative form of treatment for gynecological endocrinology dysfunctions [12–14], with significant efficacy and reduced side effects through various herbal combinations [15]. He's Yangchao Recipe (HSYC, with China Patent Application number of 201710902472X) is a special herbal prescription that originates from the ancestral experience of He's School Doctrine of Gynecology, which is one of the first studios of inheritance of academic schools of traditional Chinese medicine approved by the National Administration of TCM, and it is also the intangible cultural heritage of Hangzhou [16]. Results from previous studies of our research group have already shown that HSYC effectively increased the anti-Müllerian hormone (AMH) level and the growing follicle counts, as well as reducing serum FSH and improving ovarian reserve in patients with diminished ovarian reserve (DOR) [17, 18]. Animal experiment shows that high-dosage HSYC could notably improve ovarian reserve and alleviate the further development of DOR in mice [19].

To elucidate the potential mechanism of the therapeutic effect of HSYC, an 8-month-old C57BL/6 female mouse (represents humans at ages 38–47 according to The Jackson Laboratory) undergoing consecutive superovulation was chosen as a model to explore the regulatory effect of HSYC on protecting ovarian functions and oocytes/embryos quality after repeated superovulation.  Figure 1 shows the workflow of the study. Our results demonstrated that consecutive superovulation can compromise oocyte quality and embryo development competence, increase oxidative stress and granular cell apoptosis along with damaging mitochondrial functions, but these detrimental effects from the oxidative insult were attenuated by HSYC, probably involving ROS/JNK/P53 signaling pathway.

## 2. Materials and Methods

### 2.1. He's Yangchao Recipe

The HSYC recipe used in this study was provided by the Department of Pharmacy, Hangzhou Hospital of Traditional Chinese Medicine, and authenticated by Zhejiang University of Traditional Chinese Medicine. After the material herbs of HSYC being soaked for 30 min, HSYC was decocted with distilled water and heated for 1 h after boiling, and the mixture was then filtered. HSYC was concentrated with rotary evaporators, boiled into a thick slurry, and then was sealed and refrigerated at −20°C for later use. HSYC consists of eight traditional Chinese herbs (Table 1) as follows: 10.3% *Paeonia lactiflora* Pall; 15.5% *Cuscuta chinensis* Lam; 15.5% *Cistanche salsa* (C.A.Mey.) Beck; 10.3% *Angelica sinensis* (Oliv.) Diels; 15.5% *Rubus chingii* Hu; 12.4% Pueraria lobata (Willd.) Ohwi; 10.3% *Asparagus cochinchinensis* (Lour.) Merr; and 10.3% *Platycladus orientalis* (Linn.) Franco.

### 2.2. UPLC-ESI-MS/MS

Mix the samples with vortex after thawing and 1000 ul of them was centrifuged (12000 r/min, 4°C) for 10 min, and then filtered and stored in a sample flask. UPLC-ESI-MS/MS implement conditions are as follows: the column involved in UPLC was Agilent SB-C18 (1.8 *μ*m, 2.1 mm *∗* 100*∗*mm); pure water and 0.1% formic acid mobile phase was used for solvent *A*, and acetonitrile with 0.1% formic acid for solvent *B*; A gradient program starts with conditions under 95% *A*, and 5% *B* and lasted for 9 min, and subsequently, a linear gradient was programmed to 5% *A*, 95% *B* and lasted for 1 min. The ratio of the *B* phase is reduced to 5% again in 10.00–11.10 min and remained for 14 min, and then the effluent was connected to an ESI-Q TRAP-MS; AB4500 Q TRAP UPLC/MS/MS system was used to acquire triple quadrupole (QQQ) scans; Analyst 1.6.3. software (AB Sciex) was used to analyze the results.

### 2.3. Animals and Ethical Approval

Sixty 8-month-old female C57BL/6 mice (28–33 g), together with five nine-week-old male mice (18–20 g) for in vitro fertilization, were purchased from Beijing Charles River Laboratory Animal Company (Certificate No. SCXK 2019-0009, Beijing, China). Mice were housed in a barrier facility at the Animal Experimental Research Center of Zhejiang Chinese Medical University with constant temperatures, humidity, and daylight (12 hours light/12 hours darkness). All of the experimental procedures were supervised by the Institutional Animal Care and Use Committee of the Zhejiang Chinese Medical University (Approval number: IACUC-20201123-01), and the research was conducted in accordance with ARRIVE guidelines [20].

### 2.4. Repeated Superovulation Procedures

The 8‐month‐old female mice were randomly separated into four groups. R4 mice were the ones that underwent four superovulatory cycles. In addition, R4 mice taking N-acetyl-L-cysteine (NAC) (Sigma-Aldrich, St. Louis, USA) were termed as NR4 mice, and the remained ones taking traditional Chinese herbal prescription HSYC were termed as TR4 mice. The selection for dosage of NAC and HSYC was based on the dosage used in clinical trials and conversion of human to mouse dose. NAC dosage was determined to be 870 mg/kg [21] and 29.1 g/kg for HSYC [19] via intragastric administration daily. A dose of 10 IU of pregnant mare serum gonadotropin (PMSG; Nanjing Aibei Biotechnology Company, Nanjing, China) was administered to the female mice for repeated superovulation, followed 48 h later by 10 IU of human chorionic gonadotropin (HCG; Nanjing Aibei Biotechnology Company, Nanjing, China) every other week for 4 weeks. Mice injected with PMSG only once were set to be *R*1 mice.  Figure 2 shows the superovulation injection protocols in the present study.

### 2.5. Oocyte Collection, *In Vitro* Fertilization, and Embryo Culture

After the female mice were sacrificed by CO_2_ inhalation, the ampulla of the oviduct was obtained and placed in a test tube containing Hepes buffer, and the bulge of the ampulla of the oviduct was cut through with the needle to allow the cumulus-oocyte complexes (COCs) to slide out. The COCs from 9 mice per group were placed into the prepared Hepes containing hyaluronidase, and the number and morphology of oocytes were observed under the Stereo Microscope after 5–10 minutes of digestion. These oocytes were then collected for the subsequent experiments. The COCs from another 6 mice per group were placed in HTF fertilized drop in an incubator. The eggs were picked up and washed after 6 hours, moved to the M2 medium with mineral oil, and put into an incubator containing 5% CO_2_, whose temperature was set to 37°C, and continue to culture. Observe and record the condition of embryos at 0.5 d, 1.5 d, and 3.5 d, respectively. In addition, ovaries were collected in cryopreservation tubes, placed into liquid nitrogen, and then transferred to −80°C for future analysis.

### 2.6. ROS Assessment

Intracellular ROS levels were evaluated by the dichlorodihydrofluorescein diacetate (DHFC-DA) probe method. Oocytes were incubated with 10 mM DHFC-DA (Beyotime Biotechnology, Shanghai, China) in PBS for 20 minutes at 37°C in a dark interior. Images were captured by an inverted fluorescent microscope (Zeiss Axio Observer.A1).

### 2.7. Enzyme-Linked Immunosorbent Assay (ELISA)

The levels of serum estrogen, progesterone, and INH-B were detected using the ELISA kits (Vankew, Shanghai, China), as instructed by the manufacturer.

### 2.8. Histopathology and Electron Microscopy

The ovary tissues were fixed in 4% paraformaldehyde after mice were sacrificed and then went through paraffin embedding and serial sections. 4 *μ*m thick ovary sections were stained with hematoxylin and eosin (*H* & *E*) on a glass slide. Images of the ovaries' structure and follicles counts were taken by microscope (Motic AE2000). Immediately after dissection, the ovary tissue was fixed with glutaraldehyde and osmic acid, dehydrated, and transferred to a resin mixture. 100 nm thick ovary sections were stained with uranyl acetate and lead citrate. Images were photographed by transmission electron microscope (HITACHI-H7650).

### 2.9. TUNEL Staining of Ovarian Cells

Apoptosis of ovarian granulosa cells was observed by a One-Step TUNEL Apoptosis Assay Kit (Beyotime Biotechnology, Shanghai, China). The paraffin sections of ovaries were digested with proteinase K for 30 min and then incubated in a TUNEL test reagent composed of enzyme terminal deoxynucleotidyl transferase (TdT) and fluorescein-dUTP for 1 h in a dark interior at 37°C, and mounted in fluorescence decay-resistant medium containing DAPI. The digital images were recorded using a fluorescence microscope (Leica DM2500B).

### 2.10. Protein Expression Analysis

To extract the total protein from the mice's ovarian tissues, we used a total protein extraction reagent (KeyGen Biotech, Jiangsu, China) according to the manufacturer's protocol. The protein concentration was assayed using the BCA Protein Assay kit (KeyGen Biotech, Jiangsu, China). The Simple Western (WesProteinSimple, San Jose, CA, USA) system was used for protein quantification (JNK, Bax, and p53). The antibodies used in the above protein determination are all from Cell Signaling Technology (CST, Danvers, MA, USA). Then, the signal intensities were quantified and analyzed using Compass Software (ProteinSimple).

### 2.11. Real-Time PCR

RNA samples were prepared using TaKaRa MiniBEST Universal RNA Extraction Kit (TaKaRa, Shiga, Japan), and a reverse transcriptase reaction was performed using PrimeScript RT Master Mix (TaKaRa, Shiga, Japan). SYBR Premix Ex TaqTM II (Perfect Real Time) (TaKaRa, Shiga, Japan) was used for the detection of the specified genes. The conditions for the reverse transcription reaction are as follows: 37°C 15 min⟶85°C 5 s⟶4°C. The reverse transcription reaction system was added to tubes used for fluorescence quantitative reaction, and the amplification reaction conditions are as follows: predenaturation: 95°C 3 min; 40 cycles (95°C 10 s, 60°C 30 s); dissolution curve: starting from 55°C, increasing by 0.5°C each 30 s until 95°C, and circulate once. All reaction information is collected by ABI StepOnePlus™ Real-Time PCR System, and normalized expression was calculated as relative fold change using the formula 2^−ΔΔCT^.  Table 2 shows the primer sequences used in the quantitative real-time PCR experiment, and *β*-actin was considered as the internal reference gene.

### 2.12. Statistical Analysis

The experimental data were analyzed by Prism GraphPad software, and all results were indicated by mean ± SD. One-way analysis of variance (ANOVA) was used to analyze differences among the groups. *P* values < 0.05 were commonly considered to be statistically significant, and the number of asterisks indicates the following levels of statistical significance: ^*∗∗*^*P* < 0.01, ^*∗*^*P* < 0.05.

## 3. Results

### 3.1. The Main Bioactive Components in HSYC by LC-QQQ-MS

LC-MS was implemented to identify the main bioactive components in HSYC, and qualitative analysis was performed to elucidate the components of the HSYC based on secondary spectrum information and the local database MWDB (Metware database). As shown in Table 3, Figures 3 and 4, the main active substances are daidzein, kaempferol, astragalin, hyperin, genistein, rutin, ellagic acid, acteoside, gallic acid, Z-ligustilide, quercetin, nicotiflorin, echinacoside, paeoniflorin, ferulic acid, apigenin, puerarin, calycosin, and trillin.

### 3.2. HSYC Improves Reproductive Endocrinology Dysfunction in Mice

Superovulation following decreased ovarian function is usually accompanied by decreased levels of estrogen, progesterone, and INH-B, as is shown by the difference between groups *R*1 and *R*4 in Figure 5. However, HSYC regulated hormone levels, with progesterone, estrogen, and INH-B levels increased (*P* < 0.05).

### 3.3. HSYC Reduces ROS Levels in Oocytes of Repeated Superovulation Mice

We examined oocytes' ROS levels retrieved from the oviduct and observed that R4 oocytes had dramatically higher ROS levels than R1 oocytes (*P* < 0.01), while ROS levels were significantly reduced in HSYC-treated oocytes and NAC-treated oocytes (*P* < 0.01; Figures 6(d) and 6(e)). The above results suggest that consecutive superovulation increased ROS levels while HSYC administration could resist oxidative stress.

### 3.4. HSYC Increases the Quantity and Quality of Oocytes

We observed the oocytes retrieved from oviducts under the microscope to determine whether HSYC could influence the quantity and quality of oocytes (Figure 6(a)). As shown in Figure 6(b), fewer eggs per oviduct from superovulated mice were retrieved compared to the *R*1 group (*P* < 0.01), but HSYC could increase the egg counts (*P* < 0.01). We also evaluated the effects of HSYC treatment on oocyte quality in mice after application of HSYC for one month, and the proportions of fragmented oocytes were markedly decreased in HSYC-treated mice and NAC-treated mice compared to the *R*4 group (*P* < 0.01, Figure 6(c)).

### 3.5. HSYC Treatment Ameliorated the Histological Changes in Ovaries

We observed pathologic changes in the ovary to elucidate the mechanism by which the number of ovulated oocytes increased by HSYC after superovulation. Contrary to the *R*4 group, significantly increased numbers of developing follicles were observed in the HSYC group as well as the total follicles (Figure 7(d)). While the number of the corpus luteum increased in all three groups after the fourth cycle of ovulation compared to the *R*1 mice, it showed a more significant incline in the TR4 group (*P* < 0.01) than in the NR4 group (*P* < 0.05) (Figure 7(b)). Hemorrhagic corpus luteum, characterized by corpus luteum infiltrated with erythrocyte, was occasionally observed in ovaries in the present study, presumably indicating recent ovulation (Figure 7(a)). However, there was no difference in the percentage of Hemorrhagic CLs in the prevalence of this phenotype among the four groups (Figure 7(c)). Administration of HSYC had a considerable effect on the histological changes in the ovary during repeated ovulation.

### 3.6. HSYC Improved the Mitochondrial Morphology in Ovary

We use electron microscopy to view ultrastructural changes in the ovaries (Figures 8(a)–8(i)). What we observed is that there were marked differences among four groups in mitochondrial morphology. In the *R*1 group, most of the mitochondria were normal, the structures of which were regular, round, oval, or rod-shaped, with clear and complete crista, nevertheless mitochondria of granulosa cells in ovaries suffering from superovulation showed abnormal and damaged structures, being swollen and ruptured with aggregation, extrusion, and fusion, with cristae being vacuolated and barely visible. The percentage of abnormal mitochondrial (mitochondria with vague cristae and vacuolated mitochondria) of the TR4 group is significantly declined than the *R*4 group (*P* < 0.05, Figures 8(j) and 8(k)).

### 3.7. A Positive Effect of HSYC on Reducing Cell Apoptosis

The percentage of apoptotic granulosa cells in the antral follicles of ovaries after consecutive superovulation was estimated in the four groups (Figure 9(a)). TUNEL-positive cells occurred more in the *R*4 group than in the *R*1 group, suggesting the aggravation of apoptosis due to ovarian hyperstimulation, whereas HSYC significantly decreased the percentage of TUNEL-positive cells (*P* < 0.05, Figure 9(b)). HSYC showed a positive effect on the reduction of ovarian cell apoptosis of HSYC.

### 3.8. HSYC Inhibited JNK and p53 mRNA Expression

The JNK and p53 mRNA increased significantly in the *R*4 group versus that in the *R*1 group, while HSYC could reduce the JNK and p53 mRNA expression, as well as NAC, did (*P* < 0.05, Figures 10(b) and 10(c)). HSYC did not show a capacity in affecting the BAX mRNA expression while NAC did (*P* > 0.05, Figure 10(d)).

### 3.9. HSYC Inhibited JNK and p53 Protein Expression

Consecutive superovulation in the *R*4 model group significantly increased JNK (46 kDa) and p53 expression in the ovary compared to the *R*1 group. However, HSYC significantly decreased JNK (46 kDa) and p53 protein expression compared with the *R*4 group, as presented in Figures 10(f) and 10(g) (*P* < 0.05). The results above measured by WES are consistent with the mRNA expression measured by RT-PCR. Nevertheless, the JNK (54 kDa) and BAX protein expressions did not show significant statistical differences among the four groups (Figures 10(e) and 10(h)). Representative band images of the target proteins are shown in Figure 10(a).

### 3.10. HSYC Improved on Developmental Potential of Embryos

As shown in Figure 11, repeated superovulation resulted in a significant decline in embryos quantity obtained after four superovulation cycles, and the number of zygotes obtained from mice COCs after in vitro fertilization was markedly higher in TR4 than that in the *R*4 group (*P* < 0.05), whereas NR4 group has a more significant higher zygote count than in the *R*4 group (*P* < 0.01). The number of 2-cell stage embryos retrieved from the TR4 mice is as well higher than that in the *R*4 group (*P* < 0.05). The difference between the morula counts of the TR4 group and the *R*4 group showed statistical significance (*P* < 0.05). Embryos from mice subjected to four superovulation cycles with HSYC treated had a higher hatching potential compared with all other groups without HSYC administration.

## 4. Discussion

The aging phenomena can be attributed to increased ROS levels and accumulated oxidative damage in somatic cells and the affection of oxidative stress to oocytes has been well-demonstrated [5, 22, 23]. ROS are not only constantly generated but also eliminated in the mitochondria thus maintaining redox balance and homeostasis, and when the redox balance is broken due to aging, ROS are accumulated [24]. Mitochondria, which is crucial for controlling cell survival and death, is the most remarkable target of ROS. The accumulation of spontaneous mitochondria damage was due to increased ROS in oocytes, and mitochondria dysfunction would induce chromosomal nondisjunction, pregnancy loss, or decreased embryo viability [5, 6].

Previous studies have suggested that consecutive superovulation can harm fertility and fecundity in mice, whose AMH expressions, along with the concentrations of estrogen and progesterone significantly decreased [25]; Results of recent studies also suggest that multiple superovulations affect mitochondrial function in cumulus cells, inducing apoptosis and mitochondrial DNA (mtDNA) damage as well as altering histone modifications in early embryos, so as to decrease ovarian functions, reduce the oocyte and embryo quality and delay embryonic development [8–10]. Increased cytoplasmic fragmentation, abnormal mitochondrial distribution, and spindle damage were also observed in oocytes ovulated from mice that underwent superovulation [26]. And to be more precise, it seems that repeated superovulation induces strong oxidative stress and damage to all reproductive organs of female mice, which results in subsequent negative effects mentioned above [27, 28]. Women of late childbearing age ovulate fewer eggs beyond a loss of ovarian reserve [29]. Meanwhile, there are often difficulties for these women to respond to ovarian stimulation when undergoing IVF [30], and when pregnancy does occur to them, they will have a higher incidence of aneuploid blastocysts and unexplained recurrent abortion [31].

In this present study, we can see that as previously reported, consecutive superovulation in aged mice caused the declined serum estrogen, progesterone, and INH-B expressions, followed by reduced growing follicles, indicating impaired ovarian functions. Aging together with superovulation, contributes to the oxidative stress and ROS accumulation in the ovary, leading to the dysfunction of mitochondria of granulosa cells and the accelerated apoptosis in ovarian cells. Increased oocyte cytoplasmic fragmentation has also been observed. As is demonstrated by some research, the average number of ovulated oocytes of 4-week-old female C57BL/6 mice undergoing superovulation could reach to 42.7, while the mice aged 8 months (30 weeks) could only ovulate 16.2 oocytes [32]. Although the number of follicles after super-stimulation in 8-month-old mice is less than that of mice at their young age, the condition of continuous super-stimulation reduces ovulation simultaneously.

In contrast to the model group without drug intervention, the results of the present study revealed the efficacy of HSYC in improving ovarian function, fertility, and embryonic development. Under oxidative stress, HSYC lessened the apoptotic rate of granulosa cells (GCs) and the ROS Level of oocytes, along with an escalation in serum hormone expressions and growing follicles in ovaries. The normal morphological rate of mitochondria also increased, followed by the enhanced embryonic development potential. The Corpus luteum of the three groups after 4 times super-stimulation increased greatly, resulting in an augment in ovarian volume, while the amount of corpus luteum in the TR4 group was significantly larger than that in the *R*4 group, which may be due to the exhausted ovarian reserve after *R*4 group experienced 4 hyperstimulation without in time intervention, and we can draw this conclusion from the different ovulated follicle counts between *R*4 group and TR4 group.

The c-jun N-terminal kinase (JNK) has a necessarily close connection with oxidative damage close [33]. It has been well-demonstrated that ROS are potent inducers of JNK, and there are some studies suggesting that the proapoptotic effect of JNK activation in ROS-mediated apoptosis is closely related to the mitochondrial pathway and the p53 pathway. As is shown in the present study, the increased JNK and P53 mRNA along with corresponding proteins expression induced by ovarian super-stimulation and aging are all attenuated by HSYC. Meanwhile, JNK could mediate mitochondrial translocation of the proapoptotic gene BAX and thus activate proapoptotic Bcl-2 family members [34]; nevertheless, the change of BAX expression among *R*4, NR4, and TR4 groups did not show statistical significance in this present experiment.

The main components of HSYC have a long history of application in the historical process of traditional medicine. *Cuscuta chinensis Lam* is used for kidney tonifying and could prevent habitual abortion and improve excessive cold in female reproductive organs [35]. *Pueraria lobata (Willd.) Ohwi* exhibits phytoestrogen-like activities, regulates the endocrine system, and has beneficial effects on menopausal metabolic dysfunction due to the high levels of isoflavones it contains [36]. Danggui, the name of which in English is *Angelica sinensis* (*Oliv*.) *Diels*, is used to invigorate the blood circulation in menstrual disorders [37], while Baishao (*Paeonia lactiflora Pall*) is used to nourish blood and regulate menstruation according to the basic theory of TCM. Danggui–Baishao, which is recognized as an herb pair, is used to nourish blood and can significantly enhance the proliferation of granulosa cells in rat ovaries [38]. And research shows that TCM treatment involving kidney tonifying and blood activating methods has been proven effective in patients with primary ovarian insufficiency (POI) [39].

Bioactive compounds in traditional Chinese medications are rich in antioxidants, mainly including flavonoids, phenols, and polysaccharides. Flavonoids are potent antioxidants protecting plants from unfavorable environmental conditions [40]. Furthermore, HSYC is a great source of flavonoids, which act as antioxidants and regulate ROS homeostasis [41]. The main component are as follows: daidzein, kaempferol, astragalin, hyperin, genistein, rutin, ellagic acid, acteoside, gallic acid, Z-ligustilide, quercetin, nicotiflorin, echinacoside, paeoniflorin, ferulic acid, apigenin, puerarin, calycosin, and trillin.

Daidzein, Astragalin, Hyperin, and Genistein could lift the estrogen and progesterone levels of rats with impaired ovarian function. Moreover, Daidzein could elevate total antioxidant capacity in rats, attenuate ROS-induced toxicity by antioxidant action in ovarian cells [42, 43]; Kaempferol could maintain follicular survival, increase active mitochondria levels, prevent the H_2_O_2_-induced compromise of mitochondrial membrane potential (MMP) and ROS generation [44, 45]. Astragalin could enhance ovarian reserve and reduce ovarian GCs apoptosis in aged female rats via the Bcl-2 relative pathway [46]. Hyperin could increase proliferation and cell viability in H_2_O_2_ stimulated GCs, reverse the increased MDA level and decrease SOD, GSH-Px, and CAT, thus frequently used Chinese herbs like *Cuscuta Chinensis* Lam which contain Hyperin could improve ovarian functions through these effects [47, 48]. Genistein has antioxidant activity against radiation-mediated oxidative stress and Cyclophosphamide-induced ovarian toxicity through improving ovarian histology and immunostaining of ovarian iNOS, thus reversing ovarian apoptosis [49, 50], and meanwhile, it could elevate MMP of GCs, followed by a decline in the levels of intracellular mitochondrial superoxide and the apoptotic rate [51]. Ellagic acid could revoke ROS by manipulating oxidative biomarkers within the ovarian cells and exhibits a significant antioxidant capacity in aging and could protect the embryo DNA and development from the oxidative insult [52, 53]. The addition of acteoside during in vitro maturation could improve the rate of blastocyst formation Improve and mitochondrial morphology with decreased ROS level [54, 55]. Acteoside could also attenuate the drop of the MMP in the Chinese hamster ovary cell line (CHO) treated with H_2_O_2_ [56]. Rutin treatment before cisplatin could reduce apoptosis to preserve the normal follicles, decrease ROS levels, increase GSH levels and enhance mitochondria functions in ovaries. Rutin could also ameliorate the ischemia-reperfusion (I/R)-induced ovarian injury in rats via its possible antioxidative effects [57, 58]. Gallic acid could restrain granulosa cells apoptosis by inhibiting the expression of proapoptotic genes in mouse ovaries [59].

The relative comparative advantage of TCM compared to modern medicines is that TCM stresses compatibility, and the bioactive components in TCM act via multiple targets, while the mode of modern medicines is “one drug for one target” [60]. HSYC can not only resist oxidative stress and improve ovarian function but also regulate hormone levels. From the perspective of TCM theory, HSYC could tonify the liver and kidney, nourish essence and blood, soften the liver and benefit heart Qi, regulating body functions with a holistic concept. While resisting oxidative stress, it also improves symptoms such as insomnia, lassitude, nervousness, hot flashes, and night sweats. Herein, HSYC takes effect through multiple targets and multiple links, highlighting the unique advantages of Chinese traditional medicine.

## 5. Conclusions

The fertility of aging mice decreases and repeated superovulation could cause oxidative stress to damage ovarian function, and further reduce the number and quality of eggs. The LC-MS results indicate that HSYC contains ample and certain antioxidant bioactive compounds. The present study revealed that the TCM formula, HSYC, has exerted promising effects in promoting ovarian reserve, oocyte quality, and embryo hatching potential, and could reverse the deleterious effect induced by both aging and consecutive ovarian superovulation, potentially via the ROS/JNK/p53 pathway.

## Figures and Tables

**Figure 1:** A workflow of this study.

**Figure 2:** The superovulation treatment protocol in the present study.

**Figure 3:** MRM chromatograms in (a) negative and (b) positive modes. Identification: 1, daidzein; 2, kaempferol; 3, astragalin; 4, hyperin; 5, genistein; 6, rutin; 7, ellagic acid; 8, acteoside; 9, gallic acid; 10, Z-ligustilide; 11, quercetin; 12, nicotiflorin; 13, echinacoside; 14, paeoniflorin; 15, ferulic acid; 16, apigenin; 17, puerarin; 18, calycosin and 19, trillin.

**Figure 4:** The product ion scan spectra of 19 bioactive compounds in HSYC.

**Figure 5:** The effect of HSYC on improving reproductive endocrinology dysfunction. (a–c) The serum content of estrogen, progesterone, and INH-B level of mice in different groups, respectively.

**Figure 6:** Effect on the quantity and quality of oocytes ovulated into the oviducts of HSYC (a–c) and different ROS levels in oocytes from mice undergoing repeated superovulation with or without intervention (d, e). (a) Representative images of morphologically normal and fragmented oocytes. White arrow: oocytes with obvious cytoplasmic fragments. (e) Representative fluorescence images of ROS; scale bars are 50 *μ*m. (b) Graph showing the proportion of morphologically abnormal and fragmented oocytes in different groups. (c) Graph showing the average number of oocytes ovulated per mouse (*n* = 9 per group, 18 oviducts). (d) Quantitative fluorescence intensities of ROS staining in oocytes from the *R*1 (*n* = 32), *R*4 (*n* = 36), NR4 (*n* = 38), and TR4 (*n* = 42) groups, and n denotes the number of oocytes for each group. ROS: reactive oxygen species.

**Figure 7:** Effect on follicles after 28 days of HSYC administration. (a) Follicles observed after *H* & *E* staining. PF: primary follicles; GF: growing follicles; AF: atretic follicles.CL: corpus luteum. White arrow: hemorrhagic CLs. Scale bars, 500 *μ*m and 200 *μ*m. (b, c) The number of CLs and the percent of hemorrhagic CLs in each group. (d) The numbers of follicles at different developmental stages of maturation.

**Figure 8:** Effect on ultrastructural changes of the ovarian granulosa cells of HSYC. (a–e) Normal ultrastructure in control group mice ovaries. (f–i) Representative images of mitochondria around the granulosa cells in each group, (f) *R*1 group, (g) *R*4 group, (h) NR4 group, and (i) TR4 group. (G: golgi complex; L: lipid; M: mitochondrial; N: nucleus of granulosa cells; white arrow: abnormal mitochondria; red arrow: vacuolated mitochondria). (j, k) The percentage of mitochondria with vague cristae and vacuolated mitochondria in all mitochondria.

**Figure 9:** Effect of HSYC on ovarian cell apoptosis. (a) Apoptotic nuclei and total nuclei show green and blue fluorescence respectively. Scale bar: 500 *μ*m. (b) The percentage of TUNEL-positive granulosa cells in the antral follicles.

**Figure 10:** The effects of HSYC on superovulation-induced changes of protein JNK, p53, BAX, and mRNA levels of JNK, p53, and BAX. (a) Representative band images of the three proteins, JNK, P53, and BAX. (e–h) Relative protein levels of JNK, P53, and BAX. (b–d) Relative mRNA expression levels of JNK, P53, and BAX. The data represent at least three independent experiments.

**Figure 11:** Effect on the quality and quantity of embryos of HSYC. (a) Representative images of embryos, were acquired on 0.5 D, 1.5 D, and 3.5 D in vitro embryo culture. The red arrow indicates two-cell stage embryos, and the black arrowhead refers to morula. Scale bars = 50 *μ*m. (b) The total amount and the average number of embryos at different stages in each group.

**Table 1:** Composition of HSYC.

Chinese name	English name	Family	Plant part	Crude herb (g)
Baishao	*Paeonia lactiflora* pall	Paeoniaceae	Root	10
Tusizi	*Cuscuta chinensis* lam	Convolvulaceae	Seeds	15
Roucongrong	*Cistanche salsa* (C.A.Mey.) beck	Orobanchaceae	Stem	15
Danggui	*Angelica sinensis* (Oliv.) diels	Apiaceae	Root	10
Fupenzi	*Rubus chingii* Hu	Rosaceae	Fruit	15
Gegen	*Pueraria lobata* (Willd.) Ohwi	Leguminosae	Root	12
Tiandong	*Asparagus cochinchinensis* (Lour.) Merr.	Asparagaceae	Root	10
Baiziren	*Platycladus orientalis* (Linn.) Franco	Cupressaceae	Seed	10

**Table 2:** Primer sequences of the target genes.

Gene	Primer	Sequences(5′ to 3′)
JNK	Forward primer	AGTGACAGTAAAAGCGATGGTC
	Reverse primer	AGCACAAACAATTCCTTGGGC

p53	Forward primer	CCCCTGTCATCTTTTGTCCCT
	Reverse primer	AGCTGGCAGAATAGCTTATTGAG

Bax	Forward primer	TGAAGACAGGGGCCTTTTTG
	Reverse primer	AATTCGCCGGAGACACTCG

*β*-Actin	Forward primer	CATCCGTAAAGACCTCTATGCCAAC
	Reverse primer	ATGGAGCCACCGATCCACA

**Table 3:** The RT, MW, MS-MS fragment ions, DP and CE of HSYC.

Component	Classification	Precursor ion (*m*/*z*)	Product ion (*m*/*z*)	MW (Da)	Ionization model	DP (V)	CE (eV)	RT (min)
Daidzein	Isoflavones	255.07	137.00	254.06	[M + H]+	40	40	4.94
Kaempferol	Flavonols	285.04	151.00	286.05	[M − H]−	-40	-30	5.72
Astragalin	Flavonols	449.11	287.06	448.10	[M + H]+	50	30	4.14
Hyperin	Flavonols	463.09	300.00	464.10	[M − H]−	-60	-40	3.88
Genistein	Isoflavones	271.06	215.07	270.05	[M + H]+	20	40	5.65
Rutin	Flavonols	609.15	301.00	610.15	[M − H]−	-40	-40	3.75
Ellagic acid	Tannin	301.00	185.02	302.01	[M − H]−	-60	-40	3.89
Acteoside	Phenolic acids	623.20	461.17	624.21	[M − H]−	-50	-30	4.03
Gallic acid	Tannin	171.03	107.01	170.02	[M + H]+	50	30	1.79
Z-Ligustilide	Others	191.11	117.07	190.10	[M + H]+	20	20	8.26
Quercetin	Flavonols	303.05	137.02	302.04	[M + H]+	50	50	5.08
Nicotiflorin	Flavonoid	593.15	285.04	594.16	[M − H]−	-50	-30	4.00
Echinacoside	Phenolic acids	785.25	623.20	786.26	[M − H]−	-50	-50	3.33
Paeoniflorin	Monoterpenoids	479.16	121.03	480.16	[M − H]−	-50	-30	3.64
Ferulic acid	Phenolic acids	193.05	134.01	194.06	[M − H]−	-20	-20	4.12
Apigenin	Flavonoid	271.06	153.01	270.05	[M + H]+	50	30	5.63
Puerarin	Isoflavones	417.12	297.07	416.11	[M + H]+	50	30	3.19
Calycosin	Flavonoid	285.08	225.06	284.07	[M + H]+	50	30	5.24
Trillin	Steroidalsaponins	577.37	271.21	576.36	[M + H]+	50	30	4.75

MW: molecular weight, DP: declustering potential, CE: collision energy, and RT: retention time.

## Data Availability

The data used to support the findings of this study are included within the article.
